The article "Medical and Health Data Classification Method Based on Machine Learning" was published in 2021. Journal: J Healthc Eng.

# Medical and Health Data Classification Method Based on Machine Learning

**DOI:** 10.1155/2021/2722854

**Published:** 2021-11-16

**Authors:** Yu Zeng, Fuchao Cheng

**Affiliations:** College of Computer Science, Chengdu University, Chengdu 610106, China

## Abstract

The information defined in medical health data is researched based on machine learning-related algorithms. Also, this paper used random forest and other related algorithms to perform health data training and fitting. Research shows that the algorithm proposed in the paper can improve the progress of health data classification. The algorithm can provide technical support for the improvement of medical data classification.

## 1. Introduction

With the development of China's medical industry, the medical market has become more and more complicated. Establishing a sound medical credit system is one of the important means to regulate the medical market. The lack of standard measures for participants in China's medical market has led to frequent breaches of trust, such as registration breaches [1]. This seriously wastes limited medical resources. This article studies the dishonesty behaviour in medical treatment. The purpose of the research is to increase the medical industry's management of market participants and improve the market access threshold and management level. In recent years, the development of computer technology has made great progress in data mining and machine learning technology. Supporting massive amounts of data and using machine learning algorithms to utilize the data effectively can enhance the value of data. When the scenario of the algorithm is in the medical field, the relevant historical behaviour data of medical market participants can be used to predict whether there is a risk of dishonesty. This assists medical market managers in making decisions.

This paper studies the decision tree and random forest algorithm. Since the random forest algorithm is based on the ensemble learning idea, it effectively avoids noise in the training data set, so there will be no overfitting phenomenon. The simulation results also show that this method performs better than logistic regression and K-nearest algorithm in identifying dishonest behaviours [2]. This has important reference significance for the establishment of the medical credit system.

## 2. Theoretical Basis

### 2.1. Decision Tree Algorithm

In recent years, decision trees have been one of the most widely used algorithms in machine learning. Compared with the neural network algorithm decision tree, it has the characteristics of flexibility and strong interpretability. Flexibility embodied in the decision tree can prune the tree structure according to the wishes of the algorithm designer and improve the algorithm's performance. Interpretability is embodied in the decision-making standard with extremely high confidence when each root node of the decision tree makes a decision. The decision tree is composed of three parts: directed edges of internal nodes and leaf nodes. The basic process is shown in Figure 1.

The article "Medical and Health Data Classification Method Based on Machine Learning" was published in 2021. Journal: J Healthc Eng.

It can be seen from Figure 1 that a classification tree can divide a data set into different classifications *C*_*i*_ using different feature dimensions *A*. When the classification tree is classified, different classification tree algorithms are based on different node classification standards [3]. Figure 1 is based on information gain. The method of defining information gain is as follows.

First, define information entropy. The definition of information entropy of data set *D* is as follows:

(1) $$\begin{array}{c} \text{Info}\left(D\right)=-\sum_{i=1}^{I}\frac{\left|C_{i}\right|}{D}\log_{2}\frac{\left|C_{i}\right|}{D}. \end{array}$$

Different features have conditional information entropy Info *A*(*D*) for D:

(2) $$\begin{array}{c} {\text{Info}}_{A}\left(\left|D\right|\right)=-\sum_{k=1}^{K}\frac{\left|C_{k}\right|}{D}\times \text{Info}\left(D_{i}\right)=-\sum_{k=1}^{K}\frac{\left|C_{k}\right|}{D}\sum_{i=1}^{I}\frac{\left|C_{ki}\right|}{D}\log_{2}\frac{\left|C_{ki}\right|}{D}. \end{array}$$

The information gain of the feature at this time is

(3) $$\begin{array}{c} \text{Gain}\left(A\right)=\text{Info}\left(D\right)-{\text{Info}}_{A}\left(\left|D\right|\right). \end{array}$$

Academically, different types of decision trees use different node decision criteria. This article also uses the Gini coefficient as the decision criterion [4]. The decision tree at this time is called CART. For multiclassification problems, when there are K different categories, mark *p*_*k*_ as the probability that the current sample is category *k*. At this time, the Gini coefficient can be defined according to the probability distribution:

(4) $$\begin{array}{c} \text{Gini}\left(p\right)=\sum_{k=1}^{K}p_{k}\left(1-p_{k}\right). \end{array}$$

When there is a sample set *D*, the Gini coefficient of the sample can be written as

(5) $$\begin{array}{c} \text{Gini}\left(D\right)=1-{\sum_{k=1}^{K}\left(\frac{\left|C_{k}\right|}{\left|D\right|}\right)}^{2}. \end{array}$$

The sample set *D* is divided into different subsets *D*_1_ and *D*_2_ according to feature A:

(6) $$\begin{array}{c} D_{1}=\left\{\left(x,y\right)\in D|A\left(x\right)=a\right\},\\ D_{2}=D-D_{1}. \end{array}$$

The Gini coefficient divided according to feature A is

(7) $$\begin{array}{c} \text{Gini}\left(D,A\right)=\frac{\left|D_{1}\right|}{\left|D\right|}\text{Gini}\left(D_{1}\right)+\frac{\left|D_{2}\right|}{\left|D\right|}\text{Gini}\left(D_{2}\right). \end{array}$$

The article "Medical and Health Data Classification Method Based on Machine Learning" was published in 2021. Journal: J Healthc Eng.

### 2.2. Integrated Learning and Random Forest

In actual engineering applications, the ability of a single decision tree is limited. The noise and outliers in the training data will cause overfitting of the decision tree, which will seriously affect the accuracy of the decision tree to classify unknown data. Therefore, pruning operations are required after the decision tree is generated. To avoid overfitting, random forest (RF) can also be used [5]. The establishment of the random forest depends on the guidance of integrated learning thought (bagging). Bagging is characterized by random sampling of samples and classifiers. It includes two steps: selecting samples for model training and classifying based on classifiers. The process is shown in Figure 2.

It can be seen from Figure 2 that the difficulty of ensemble learning lies in the random sampling of samples and the design of combining strategies between different learners. This article uses booststrapping to extract training samples *T* during random sampling. The extraction is divided into *k* rounds. After *k* rounds of extraction, *k* training sets can be obtained [6]. The probability of not being selected in the original data is

(8) $$\begin{array}{c} \underset{N->\infty }{\lim}{\left(1-\frac{1}{N}\right)}^{N}\approx 0.368. \end{array}$$

After randomly generating the training set, the decision tree is generated. K training sets can train *k* decision trees. During the training process, the decision tree does not need to be pruned. After the training is completed, *k* weak classifiers can be obtained. Then, assign the same weight to different classifiers to get a strong classifier [7]. To measure the classification performance of the random forest, we need to define the interval function of the random forest:

For the classifier {*h*_1_(*x*), *h*_2_(*x*), ⋯, *h*_*N*_(*x*)}, there is a sample set {*X*, *Y*}. Its distribution is *X*, *Y*:

(9) $$\begin{array}{c} \text{mg}\left(x,y\right)=a\upsilon_{k}I\left(h_{k}\left(x\right)=y\right)-\max_{j\neq y}a\upsilon_{k}I\left(h_{k}\left(x\right)=j\right). \end{array}$$

The interval function of the random forest algorithm can be denoted as var(mr), and its upper bound can be given by the following formula:

(10) $$\begin{array}{c} \text{var}\left(\text{mr}\right)\leq \frac{\bar{P}\left(1-s^{2}\right)}{s^{2}}. \end{array}$$

*s* represents the classification strength of a single decision tree, and *P* represents the correlation between decision trees. The above formula shows that the interval function of the random forest has an upper limit. This upper limit can be lowered when the strength of a single classification tree is increased, and the correlation between each tree is reduced.

The article "Medical and Health Data Classification Method Based on Machine Learning" was published in 2021. Journal: J Healthc Eng.

## 3. Method Implementation

### 3.1. Data Input

This article investigates the three parties of patients, hospitals, and medical companies. Then, from the patients' perspective, random forest algorithms identify dishonest behaviours to build a healthy medical platform. First of all, this article obtained data sets related to citizen credit from public data sets [8]. In the random forest training, because the privacy of medical patients is involved, the residents' credit data can only be obtained from the foreign platform Lending Club. Then, add relevant medical record information to each data to ensure that the data are suitable for the application scenarios required in this article. After the data set is collected, the data are preprocessed according to the data preprocessing process shown in Figure 3 [9].

When dealing with outliers, mainly eliminate data items that are seriously inconsistent with logic. The method used in the article is Turkey's algorithm. This method can define the data of 1.5 times the 4th quartile range as outliers according to the distribution characteristics of the data and eliminate them. The data normalization process uses the following formula:

(11) $$\begin{array}{c} \frac{\left(X-\min\left(X\right)\right)}{\max\left(X\right)-\min\left(X\right)}. \end{array}$$

After the data are normalized, the value of the data itself will not cause an offset to the evaluation result, and the evaluation result only depends on the influence of the data attribute. The final step of preprocessing is to perform correlation analysis on the data. We eliminate the more relevant attributes in the data to reduce the dimensionality of the input data under the premise of ensuring the classification accuracy, thereby improving the efficiency of model training and classification.

### 3.2. Algorithm Training and Testing

In the random forest, it is necessary to reasonably set the relevant parameters of the random forest algorithm according to the feature vector dimension and the data dimension. This paper analyzes the error of random forest under different parameters [10]. The error analysis results are shown in Figures 4 and 5.

Figures 4 and 5, respectively, show the impact of different ntry and mtry on the model's accuracy during training. For random forests, the value of ntryshould be large enough to ensure that the model can converge during the training process.  Figure 4 shows the model error under different ntry when the default mtry is mtry=sqrt(*M*). It can be seen that when ntry reaches 1000, the model error drops to a stable level.  Figure 5 shows the effect of different mtry on model accuracy when ntry=1000. It can be seen that when mtry < 6, the model error increases as mtry increases. When mtry > 6, the model error increases as mtry increases. Therefore, the optimal value of mtry is 6.

The article "Medical and Health Data Classification Method Based on Machine Learning" was published in 2021. Journal: J Healthc Eng.

In addition to mtry and ntry, the important parameters of random forests also include classes. In the subsequent model training and testing, the value of each parameter is shown in Table 1.

After setting the parameters of the model, we trained and tested the model. To better identify the efficiency of the batch model in the medical dishonesty behavior, this paper uses logistic regression (LR) and *k*-neighbor algorithm (*k*-NN) for comparison. The recognition accuracy of each algorithm is shown in Table 2.

In Table 2, the actual rate is the rate predicted by the positive model for the sample. The true negative rate is the negative rate but is predicted to be positive by the model. It can be seen from Table 2 that the actual rate of the RF algorithm is 12.9%, which is an improvement over *k*-NNLR. The accuracy rate is 1.4% and 1.3% higher than that of *k*-NN and LR, respectively. The true negative rate has dropped to a certain extent. It can be seen that the RF algorithm has better performance when recognizing unpredictable medical behaviours.

## 4. Conclusion

This article is based on the idea of machine learning and data mining to research medical and health data. The article establishes a prevention and monitoring model based on the random forest algorithm. This article focuses on the input features used in related medical models. In addition to combining the historical medical information of medical participants, we also introduce the patient's social credit status, which can effectively compensate for the behavior identification of medical record personnel and the prevention of dishonesty. The random forest algorithm used in this article can avoid the overfitting phenomenon in the training process and improve the prediction accuracy. The content of this article has certain practical significance for the behavioral norms of medical market participants.

## Figures and Tables

**Figure 1:** Decision tree algorithm flow.

**Figure 2:** Bagging algorithm flow.

**Figure 3:** Data preprocessing process.

**Figure 4:** The effect of ntry on model accuracy.

**Figure 5:** The effect of mtry on model accuracy.

**Table 1:** Random forest parameter settings.

Parameter name	Parameter description	Parameter value
Ntree	Tree of tree	1000
Mtry	Number of variables selected by the tree node	6
Class weight	Class weight	(1,50)

The article "Medical and Health Data Classification Method Based on Machine Learning" was published in 2021. Journal: J Healthc Eng.

**Table 2:** Model indicators of different algorithms.

Model	True rate (%)	True negative rate (%)	Accuracy (%)
RF	12.90	99.10	86.60
k-NN	1.60	99.40	85.20
LR	1.60	99.50	85.30

## Data Availability

The data used to support the findings of this study are available from the corresponding author upon request.
